# Ginsenoside Rg1 protects human renal tubular epithelial cells from lipopolysaccharide-induced apoptosis and inflammation damage

This article has been retracted.

**DOI:** 10.1590/1414-431X20176611

**Published:** 2017-12-11

**Authors:** X.J. Ni, Z.Q. Xu, H. Jin, S.L. Zheng, Y. Cai, J.J. Wang

**Affiliations:** Transplantation Center, The First Affiliated Hospital of Wenzhou Medical University, Wenzhou, China

**Keywords:** Ginsenoside Rg1, LPS, Apoptosis, Inflammation, PI3K/AKT pathway, NF-κB pathway

## Abstract

Ginsenoside Rg1, one of the most notable active components of *Panax ginseng*, has been widely reported to exert anti-inflammatory actions. This study aimed to reveal whether ginsenoside Rg1 also exhibits beneficial roles against lipopolysaccharide (LPS)-induced apoptosis and inflammation in human renal tubular epithelial cells, and to evaluate the potential role of the component on tubulointerstitial nephritis treatment. HK-2 cells were treated with various doses of ginsenoside Rg1 (0, 50, 100, 150, and 200 μM) in the absence or presence of 5 μg/mL LPS. Thereafter, CCK-8 assay, flow cytometry, western blot, migration assay, reactive oxygen species (ROS) assay, and ELISA were carried out to respectively assess cell viability, apoptosis, migration, ROS activity, and the release of inflammatory cytokines. As a result, ginsenoside Rg1 protected HK-2 cells from LPS-induced injury, as cell viability was increased, cell apoptosis was decreased, and the release of MCP-1, IL-1β, IL-6, and TNF-α was reduced. Ginsenoside Rg1 functioned to HK-2 cells in a dose-dependent manner, and the 150 μM dose exhibited the most protective functions. Ginsenoside Rg1 had no significant impact on cell migration and ROS activity, while it alleviated LPS-induced ROS release and migration impairment. Furthermore, the down-regulations of p-PI3K, p-AKT, and up-regulations of PTEN, p-IκBα, p-p65, Bcl-3 induced by LPS were recovered to some extent after ginsenoside Rg1 treatment. In conclusion, ginsenoside Rg1 protects HK-2 cells against LPS-induced inflammation and apoptosis via activation of the PI3K/AKT pathway and suppression of NF-κB pathway.

## Introduction

Ginseng, the root of the widely popular plant *Panax ginseng*, has been used as Chinese traditional medicine for at least 1000 years (1). Currently, it is one of the most extensively researched and prescribed alternative medicines worldwide (1). This drug exerts pharmacological actions for several diseases including diabetes, neurological condition, cardiovascular disease, and even cancer (1 [Bibr B02] [Bibr B03]–4). The molecular components responsible for the beneficial effect of ginseng include ginsenosides, which are triterpene saponins that consist of rigid steroid skeleton and sugar moieties. Among the 30 different varieties of ginsenosides, Rg1 is one of the major pharmacologically active and abundant ingredient (1). Several studies have demonstrated the different beneficial effects of ginsenoside Rg1, which include anti-inflammatory and anti-apoptotic effects (1 [Bibr B05] [Bibr B06]–7). An early *in vivo* study has reported that intraperitoneal injection with ginsenoside Rg1 in rats resulted in a prevention of urinary protein excretion, an elevation of serum cholesterol content, as well as histopathological changes such as hypercellularity and adhesion (8), indicating the therapeutic potential of ginsenoside Rg1 in nephritis. However, to our knowledge, the detailed functions of ginsenoside Rg1 on tubulointerstitial nephritis and its underlying molecular mechanisms have not been uncovered.

PI3K/AKT pathway has been shown to play a central role in different biological processes such as angiogenesis, tumorigenesis, and inflammation (3). This pathway is also known to play an important role in inflammation by taking part in cell growth modulation, and maturation of different cellular components of the inflammation pathway (3). Similarly, NF-κB pathway is responsible for modulating multiple cellular processes especially in inflammation and apoptosis (4). Several chronic inflammation diseases like inflammatory bowel disease, sepsis, arthritis, and atherosclerosis have been revealed to be associated with chronic activation of NF-κB (4,7). Recent studies have indicated that ginsenoside Rg1 is able to activate PI3K/AKT signaling through a glucocorticoid receptor (GR)-dependent manner, and it has been shown to be a functional ligand of GR (9). In contrast, ginsenoside Rg1 suppresses the activation of NF-κB pathway also through a GR-dependent manner (4,10). Based on these findings we hypothesize that ginsenoside Rg1 might be a potential anti-inflammatory drug at least in part via modulation of PI3K/AKT and NF-κB pathways.

This study aimed to explore the beneficial role of ginsenosides Rg1 against lipopolysaccharide (LPS)-induced apoptosis and inflammation damage in human renal tubular epithelial cells and also investigate its underlying mechanism. This study will provide *in vitro* information supporting ginsenoside Rg1 as a potential anti-inflammatory drug for tubulointerstitial nephritis treatment.

## Material and Methods

### Cell culture and treatment

Human renal tubular epithelial cell line HK-2 was obtained from American Type Culture Collection (ATCC, USA), and was cultured in Dulbecco's Modified Eagle's Medium/Nutrient Mixture F-12 (DMEM-F12, 3:1, Gibco-BRL, USA) supplemented with 10% fetal bovine serum (FBS, Gibco-BRL) in a humidified 5% CO_2_ atmosphere at 37°C.

Ginsenoside Rg1 with purity greater than 98% (National Institutes for Food and Drug Control, China) were dissolved in DMSO (Sigma-Aldrich, USA) and mixed with the medium so that the final concentration of the vehicle was less than 0.1%. To analyze the functional impacts of ginsenoside Rg1 following LPS stimulation, cells were incubated with various doses of ginsenoside Rg1 (0, 50, 100, 150, and 200 μM) in the presence or absence of 5 μg/mL LPS (from *Escherichia coli* O111:B4, Sigma-Aldrich) for 24 h (11).

### CCK-8 assay

The viability of HK-2 cells was assessed by using a Cell Counting Kit-8 (CCK-8, Dojindo Molecular Technologies, USA). Briefly, cells were seeded on a 96-well plate with a density of 5×10^3^ cells/well, and then cells were treated with ginsenoside Rg1 and/or LPS for 24 h. The cells were further incubated in fresh medium for 48 h, and then 10 µL CCK-8 solution was added to the culture medium. The plates were incubated for 30 min at 37°C in humidified 95% air and 5% CO_2_. The absorbance was measured at 450 nm using a Microplate Reader (Bio-Rad, USA).

### Apoptosis analysis

The FITC-Annexin V/PI detection kit from Beijing Biosea Biotechnology Co., Ltd. (China) was utilized in the present work for detection of cell apoptosis. In brief, cells were grown to about 70% confluence in 6-well plates and treated with ginsenoside Rg1 and/or LPS for 24 h, followed by 48-h incubation in fresh medium at 37°C. Cells (1×10^5^) in each sample were then collected and resuspended in 200 µL Annexin-Binding Buffer, and stained with 10 µL FITC-Annexin V and 5 µL PI for 30 min in the dark at room temperature. Flow cytometry analysis was done by using a FACS can (Beckman Coulter, USA).

### Western blot

The protein used for western blotting was extracted using RIPA lysis buffer (Beyotime Biotechnology, China) supplemented with protease inhibitors (Roche, Switzerland). The proteins were quantified using the BCA™ Protein Assay Kit (Pierce, USA). The western blot system was established using a Bio-Rad Bis-Tris Gel system according to the manufacturer's instructions. Primary antibodies were prepared in 5% blocking buffer at a dilution of 1:1,000. Primary antibody was incubated with the membrane at 4°C overnight, followed by wash and incubation with secondary antibody marked by horseradish peroxidase for 1 h at room temperature. After rinsing, the polyvinylidene difluoride (PVDF) membrane carrying blots and antibodies were transferred into the Bio-Rad ChemiDoc™ XRS system, and then 200 µL Immobilon Western Chemiluminescent HRP Substrate (Millipore, USA) was added to cover the membrane surface. The signals were captured and the intensity of the bands was quantified using Image Lab™ Software (Bio-Rad, China).

### Migration assay

Cell migration was determined by using a modified Transwell chamber with a pore size of 8 mm (Corning, USA). For migration assay, cells suspended in 200 mL of serum-free medium were seeded on the upper compartment of 24-well Transwell culture chamber, and 600 mL of complete medium containing 10 µL mitomycin C was added to the lower compartment. After 12 h incubation at 37°C, cells were fixed with methanol. Non-traversed cells were carefully removed from the upper surface of the filter with a cotton swab. Traversed cells on the lower side of the filter were stained with crystal violet (Sigma-Aldrich) and counted. Relative cell migration was calculated as the number of the treated cells normalized to the number of the control cells adhering to the lower chamber.

### Reactive oxygen species (ROS) assay

ROS was measured by flow cytometry using 2,7-dichlorofluorescein diacetate (DCFH-DA; Nanjing Jiancheng Technology Co., China). The cells were seeded in a 6-well plate, and after treatment and washing twice with phosphate buffer saline (PBS), cells were incubated in serum-free culture medium containing 10 μM DCFH-DA for 20 min at 37°C in the dark. Subsequently, the cells were washed with PBS, and a trypsin digestion method was used for sample collection. All samples were centrifuged and the supernatants were removed. The cells were resuspended to 500 µL PBS and the fluorescent intensities were measured using a flow cytometer (488 nm excitation, 521 nm emission).

### Enzyme-linked immunosorbent assay (ELISA)

Culture supernatant was collected from 24-well plates and concentrations of MCP-1, IL-1β, IL-6, and TNF-α were measured by human CCL2/MCP-1 Quantikine ELISA kit, human IL-1 beta/IL-1F2 Quantikine ELISA kit, human IL-6 Quantikine ELISA kit, and human TNF-alpha Quantikine ELISA kit (all from R&D Systems, UK), respectively, according to the manufacturer's instructions.

### Statistical analysis

All experiments were done in triplicate. The results of multiple experiments are reported as means±SD. Statistical analyses were performed using Graphpad statistical software (GraphPad Software Inc., USA). P values were calculated using one-way analysis of variance (ANOVA). P<0.05 was considered to be statistically significant.

## Results

### Ginsenoside Rg1 alleviated LPS-reduced HK-2 cells viability

HK-2 cells were treated with increasing doses of ginsenoside Rg1 (structure depicted in Figure 1A) in the presence or absence of 5 μg/mL LPS, and then cell viability was measured to evaluate the functional effects of ginsenoside Rg1 on cell viability. At doses of 100 µm (P<0.05), 150 µm (P<0.01), and 200 µm (P<0.01), ginsenoside Rg1 caused a significant increase in the cell viability compared to control group of HK-2 cells (Figure 1B). In addition, 5 μg/mL of LPS dramatically reduced cell viability (P<0.001), while 100 µm (P<0.05), 150 µm (P<0.01), and 200 µm (P<0.01) ginsenoside Rg1 partially alleviated LPS-reduced cell viability (Figure 1C).

**Figure 1.** *A*, Structural formula of ginsenoside Rg1. *B*, Viability of HK-2 cells treated with ginsenoside Rg1 (0, 50, 100, 150, and 200 μM) or pretreated with 5 μg/mL lipopolysaccharide (LPS) (*C*). Data are reported as means±SD (n=3). ^*^P<0.05, ^**^P <0.01, and ^***^P<0.001 (ANOVA).

### Ginsenoside Rg1 alleviated LPS-induced HK-2 cells apoptosis

Cell apoptosis was also detected following various doses of ginsenoside Rg1 in the presence or absence of LPS. Flow cytometry detection results showed that 5 μg/mL of LPS induced a significant increase in apoptotic cell rate (P<0.001, Figure 2A). High doses of ginsenoside Rg1 (100, 150, and 200 μM) significantly suppressed LPS-induced apoptosis (P<0.01 or P<0.001). Expression changes of apoptosis-related factors in cells were detected by western blot analysis, as shown in Figure 2B and C. Bax and p53 were up-regulated, Bcl-2 was down-regulated, while caspase-3 was cleaved after LPS stimulation (all P<0.001). More importantly, 100, 150, and 200 μM of ginsenoside Rg1 could alleviate LPS-induced abnormal expressions of these factors (P<0.05, P<0.01 or P<0.001), and it seemed that the regulatory effects of ginsenoside Rg1 might be in a dose-dependent manner.

**Figure 2.** Ginsenoside Rg1 inhibited lipopolysaccharide (LPS)-induced HK-2 cells apoptosis. HK-2 cells were treated with ginsenoside Rg1 (0, 50, 100, 150, and 200 μM) in the absence or presence of 5 μg/mL LPS, and then apoptotic cell rate (*A*), and protein expression levels of Bax, Bcl-2, p53, cleaved-caspase3, and pro-caspase3 were assessed (*B* and *C*). Data are reported as means±SD (n=3). ^*^P<0.05, ^**^P<0.01, and ^***^P<0.001 (ANOVA).

### Ginsenoside Rg1 alleviated LPS-reduced migration in HK-2 cells

To detect the role of ginsenoside Rg1 in the migration of human renal tubular epithelial cells, HK-2 cells were treated with LPS and/or 150 µm ginsenoside Rg1, and then cell migration was assessed. LPS significantly reduced the relative migration rate (P<0.001), while ginsenoside Rg1 showed no effect on the migration of HK-2 cells. Moreover, ginsenoside Rg1 at a dose of 150 µm significantly (P<0.05) suppressed LPS-induced decrease in migration of HK-2 cells (Figure 3).

**Figure 3.** Ginsenoside Rg1 alleviated lipopolysaccharide (LPS)-induced HK-2 cell migration. HK-2 cells were treated with 150 μM of ginsenoside Rg1 and/or 5 μg/mL of LPS, and then relative migration rate was detected. Data are reported as means±SD (n=3). ^*^P<0.05 (ANOVA).

### Ginsenoside Rg1 decreased LPS-induced ROS

Given that overproduction of ROS can induce apoptosis through both extrinsic and intrinsic pathways (12), we further detected ROS activity of the HK-2 cells following by treatment with LPS and/or 150 µm ginsenoside Rg1. As mean fluorescence intensity of ROS showed in Figure 4, LPS significantly (P<0.001) increased the ROS activity of the HK-2 cells compared to the control cells (HK-2 cells in absence of LPS). Ginsenoside Rg1 (150 µm) had no impact on ROS activity, while it alleviated the LPS-induced increase of ROS activity (P<0.01).

**Figure 4.** Ginsenoside Rg1 decreased lipopolysaccharide (LPS)-induced increase in reactive oxygen species (ROS) activity. HK-2 cells were treated with 150 μM of ginsenoside Rg1 and/or 5 μg/mL of LPS, and then ROS activity was detected. Data are reported as means±SD (n=3). ^**^P<0.01 and ^***^P<0.001 (ANOVA).

### Ginsenoside Rg1 decreased LPS-induced inflammation response

The concentrations of four inflammatory cytokines, MCP-1, IL-1β, IL-6, and TNF-α, in HK-2 cells culture supernatant were detected following ginsenoside Rg1 and LPS treatment. As shown in Figure 5A-D, LPS exposure significantly elevated these four inflammatory cytokines levels in HK-2 cells culture supernatants (all P<0.001). However, ginsenoside Rg1 decreased LPS-induced production of these four cytokines (P<0.05, P<0.01 or P<0.001). A high dose of ginsenoside Rg1 exhibited a stronger down-regulatory impact on these cytokines, and the maximum decrease in the levels of the above-mentioned cytokines of inflammation were seen at a dose of 150 µm.

**Figure 5.** Ginsenoside Rg1 decreased lipopolysaccharide (LPS)-induced inflammation response. HK-2 cells were treated with ginsenoside Rg1 (0, 50, 100, 150, and 200 μM) in the absence or presence of 5 μg/mL LPS, and then the concentrations of (*A*) MCP-1, (*B*) IL-1β, (*C*) IL-6, and (*D*) TNF-α in culture supernatant were measured. Data are reported as means±SD (n=3). ^*^P<0.05, ^**^P<0.01, and ^***^P<0.001 (ANOVA).

### Ginsenoside Rg1 suppressed LPS-induced HK-2 cells injury by activation of PI3K/AKT and inactivation of NF-κB signaling pathways

Further, we focused on PI3K/AKT and NF-κB signaling pathways to reveal whether they are implicated in ginsenoside Rg1 modulation of HK-2 cells. Western blot analysis showed that p-PI3K and p-AKT levels were down-regulated, and PTEN (phosphatase and tensin homolog), p-IκBα, p-p65, and Bcl-3 were up-regulated after LPS stimulation (all P<0.001, Figure 6A-D). Meanwhile, ginsenoside Rg1 recovered these down-regulations and up-regulations (P<0.05, P<0.01 or P<0.001), in a dose-dependent manner. No impact was observed in the total levels of PI3K, AKT, IκBα and p65 after LPS and/or ginsenoside Rg1 treatment.

**Figure 6.** Ginsenoside Rg1 suppressed lipopolysaccharide (LPS)-induced HK-2 cells injury by activation of PI3K/AKT and inactivation of NF-κB signaling pathways. HK-2 cells were treated with ginsenoside Rg1 (0, 50, 100, 150, and 200 μM) in the absence or presence of 5 μg/mL LPS, and then the protein expressions of p-PI3K, PI3K, p-AKT, AKT, and PTEN, (*A*), as well as the protein expressions of p-IκBα, IκBα, p-p65, p65, and Bcl-3 (*B*) were determined by western blot analysis. *C* and *D*, Quantitative analysis based on the results from *A* and *B*. Data are reported as means±SD (n=3). ^*^P<0.05, ^**^P<0.01, and ^***^P<0.001 (ANOVA).

## Discussion

Ginsenoside Rg1, the principal component of Chinese medicinal plant *Panax*, is well-known to possess several beneficial effects (1). Studies have described the protective role of ginsenoside Rg1 in diseases associated with cardiovascular system, nervous system, using umbilical cord cells and stem cells (1–7).

The most important beneficial effects of ginsenoside Rg1 include anti-apoptosis and anti-inflammatory actions. Hu and his colleagues reported that ginsenoside Rg1 protects murine stem cells against H_2_O_2_-induced apoptosis, as evidenced by the down-regulation of cleaved caspase-3 and up-regulation of Bcl-2 (5). Furthermore, it has been demonstrated that ginsenoside Rg1 protects against H_2_O_2_-induced apoptosis in a dose-dependent mechanism (13). The molecule also can inhibit the production of LPS-stimulated cytokines (10), and protect from ischemia/reperfusion injury through attenuation of inflammation and apoptosis (14,15). Similar to these studies, we also found anti-apoptotic and anti-inflammatory roles of ginsenoside Rg1 in LPS-stimulated human renal tubular epithelial cells, as HK-2 cells viability was increased, the percentage of apoptotic cell was reduced, and the production of inflammatory cytokines (MCP-1, IL-1β, IL-6, and TNF-α) were decreased following treatment with increasing doses of ginsenoside Rg1 in the presence of LPS.

It is widely accepted that relatively high levels of ROS cause redox imbalance and induce cell apoptosis or necrosis in a wide variety of physiological and pathological conditions (16,17). On the other hand, the generation of ROS can be promoted by pro-inflammatory cytokines, such as IL-1β and TNF-α, and further deteriorate the inflammation response (18,19). In the current study, we found that ginsenoside Rg1 had no significant impact on ROS activity, but significantly reduced LPS-induced ROS. This finding further confirmed that ginsenoside Rg1 exerts anti-apoptotic and anti-inflammatory roles in LPS-stimulated HK-2 cells.

In addition to the importance of cell apoptosis and inflammation, numerous other events such as cell migration play pivotal roles in the structure and function of renal tubular epithelial cells (20,21). Migration is necessary for the renal tubular epithelial cells to acquire normal morphology, cell-cell contact, and transport capacity (22,23). To date, several studies have focused on the role of ginsenoside Rg1 in cell migration, however the mechanism of the interaction is controversial. In breast cancer MCF-7 cells, ginsenoside Rg1 treatment suppress phorbol myristate acetate-induced cell migration and invasion (4). In contrast, in endothelial progenitor cells, ginsenoside Rg1 could promote cell migration in a dose- and time-dependent manner (24). The discrepancy might be due to the different cell types and stress stimuli. In this study, we found that ginsenoside Rg1 treatment had no impacts on HK-2 cells migration, while it could alleviate LPS-reduced migration, indicating a protective role in LPS-induced impairment of migration capacity. This fact revealed that ginsenoside Rg1 improves cell migration not via modulation of epithelial mesenchymal transition (EMT) process, because in that case normal cells (undamaged) treated with ginsenoside Rg1 would also acquire migration capacity enhancement. The exact mechanism of ginsenoside Rg1 effect on human renal tubular epithelial cells migration still needs further investigation.

The PI3K/AKT is an important component of the intracellular signaling pathways tightly linked with cell proliferation, apoptosis, and inflammation response (25 [Bibr B26]–27). NF-κB pathway, a family of transcription factors, is responsible for various biological processes, especially immune and inflammation responses (28,29). More interestingly, PI3K/AKT can impact on crosstalk with NF-κB pathway (30), as it is known to regulate the transcriptional activity of NF-κB pathway through phosphorylation and facilitation of IκBα degradation (28). In this study, we explored the protein expressions of main factors in this two signaling pathways and found that PI3K/AKT pathway was activated and NF-κB pathway was suppressed following ginsenoside Rg1 treatment. These data indicated the underlying mechanisms of anti-inflammatory and anti-apoptotic actions of ginsenoside Rg1. Our findings are similar to several other studies that reported that ginsenoside Rg1 activates PI3K/AKT signaling (3), and suppresses NF-κB pathway (4,7,31,32).

In conclusion, we suggest that ginsenoside Rg1 plays an important role in the protection of HK-2 cells against LPS-induced inflammation and apoptosis. PI3K/AKT and NF-κB may be two signaling pathways contributing to the protective functions of this molecule on LPS-stimulated HK-2 cells. This study provides information on the therapeutic potential of ginsenoside Rg1 in tubulointerstitial nephritis.
